# Suppressive effect of platycodin D on bladder cancer through microRNA-129-5p-mediated PABPC1/PI3K/AKT axis inactivation

This article has been retracted.

**DOI:** 10.1590/1414-431X202010222

**Published:** 2021-01-15

**Authors:** Dayin Chen, Tingyu Chen, Yingxue Guo, Chennan Wang, Longxin Dong, Chunfeng Lu

**Affiliations:** 1 Basic Medical College, Jiamusi University, Department of Pharmacology, JiamusiHeilongjiang China Department of Pharmacology, Basic Medical College, Jiamusi University, Jiamusi, Heilongjiang, China; 2 the First Affiliated Hospital of Jiamusi University, Department of Urology, JiamusiHeilongjiang China Department of Urology, the First Affiliated Hospital of Jiamusi University, Jiamusi, Heilongjiang, China; 3 Huzhou University, School of Medicine, HuzhouZhejiang China School of Medicine, Huzhou University, Huzhou, Zhejiang, China

**Keywords:** Platycodin D, Bladder cancer, microRNA-129-5p, PABPC1, PI3K/AKT signaling pathway

## Abstract

Platycodin D (PD) is a major constituent of *Platycodon grandiflorum* and has multiple functions in disease control. This study focused on the function of PD in bladder cancer cell behaviors and the molecules involved. First, we administered PD to the bladder cancer cell lines T24 and 5637 and the human uroepithelial cell line SV-HUC-1. Cell viability and growth were evaluated using MTT, EdU, and colony formation assays, and cell apoptosis was determined using Hoechst 33342 staining and flow cytometry. The microRNAs (miRNAs) showing differential expression in cells before and after PD treatment were screened. Moreover, we altered the expression of miR-129-5p and PABPC1 to identify their functions in bladder cancer progression. We found that PD specifically inhibited the proliferation and promoted the apoptosis of bladder cancer cells; miR-129-5p was found to be partially responsible for the cancer-inhibiting properties of PD. PABPC1, a direct target of miR-129-5p, was abundantly expressed in T24 and 5637 cell lines and promoted cell proliferation and suppressed cell apoptosis. In addition, PABPC1 promoted the phosphorylation of PI3K and AKT in bladder cancer cells. Altogether, PD had a concentration-dependent suppressive effect on bladder cancer cell growth and was involved in the upregulation of miR-129-5p and the subsequent inhibition of PABPC1 and inactivation of PI3K/AKT signaling.

## Introduction

Bladder cancer is the 7th and 14th most common neoplastic disease in men and women, respectively, worldwide (1). Approximately 80% of bladder cancers are considered to have relatively favorable outcomes and are termed as non-muscle invasive bladder cancer. The remaining bladder cancers are categorized as muscle invasive bladder cancer and are characterized by a distant invasive potential (2). Due to the lack of marked symptoms at early stages, most bladder cancers are not diagnosed until the affected patient reports painless hematuria. In addition to the general limitations of carcinoma diversity and treatment options, the outcomes of muscle invasive bladder cancer remain poor (3). Therefore, developing novel, less invasive, effective, and economic strategies for the treatment of bladder cancer is of great importance.

*Platycodon grandiflorus* (Jacq.) A. DC. is the sole species in the genus *Platycodon* that is broadly distributed in Northeast Asia. It has a long history of application as a conventional herbal medicine for the treatment of ailments, such as cough, phlegm, and lung abscess (4). Platycodin D (PD) is one of the primary components of *P. grandiflorum* and has been reported to have diverse pharmacological and biological activities, including antivirus, anti-inflammation, anti-atherosclerosis, anti-nociception, anti-obesity, hepatoprotective, immunoregulatory, and anti-cancer activities; its anti-cancer potential has been increasingly studied recently (5).

MicroRNAs (miRNAs), which comprise 17-25 nucleotides and represent a major class of non-coding RNAs, have a primary function in the regulation of gene expression post-transcription, and thereby have close correlations with the development of multiple diseases when they are dysregulated (6). Unsurprisingly, the aberrant expression of miRNAs is often noted in different stages of cancers, from the initiation and onset to development and progression (7); bladder cancer is no exception for such aberrant expression (8). In this study, a miRNA microarray analysis was performed, which identified that miR-129-5p was significantly increased following the PD treatment of cancer cells. Intriguingly, miR-129-5p has been identified as an RNA sponge for the long non-coding RNA ARSR (activated in renal cell carcinoma with sunitinib resistance) and was reported to promote the proliferation and metastasis of bladder cancer cells (9). This suggests that miR-129-5p may be regulated by PD, influencing the progression of bladder cancer. In addition, poly (A) binding protein cytoplasmic 1 (PABPC1), which has been identified as one of the nine HUB nodes linked to the molecular networks specific for kidney, bladder, and prostate cancers (10), was recognized as a target mRNA of miR-129-5p in the present study. Based on these findings, we hypothesize that PD treatment suppresses bladder cancer progression, potentially through the involvement of miR-129-5p. We performed experiments on two cancer cell lines, T24 and 5637, to validate our hypothesis and to identify the potentially underlying mechanisms.

## Material and Methods

### PD preparation

PD (PunChem CID: 162859) was purchased from Yuanye Biotechnology Co., Ltd. (China). A stock solution of PD was prepared by dissolving it in DMSO (Sigma Chemical Co., Ltd., USA) to a concentration of 40 mM; the solution was stored at -20°C until use.

### Cell culture

Bladder cancer cell lines T24 (ATCC^®^ HTB-4™) and 5637 (ATCC^®^ HTB-9™) and human uroepithelial cell line SV-HUC-1 (ATCC^®^ CRL-9520™) were acquired from ATCC (USA). The cells were cultured in Roswell Park Memorial Institute (RPMI)-1640 medium (Gibco, USA) that was supplemented with 10% fetal bovine serum (FBS) and 100 U/mL penicillin-streptomycin and incubated at 37°C in a humidified atmosphere containing 5% CO_2_.

### Cell transfection

The PABPC1 sequence was synthesized and sub-cloned into a pcDNA3.1 vector (pcDNA-PABPC1, Invitrogen, USA) by GenePharma Co., Ltd. (China), and the pcDNA3.1 empty vector (pcDNA) was used as a control. miR-129-5p mimic, miR-129-5p inhibitor, the corresponding negative controls (NC), and the small interfering (si) RNAs of PANPC1 (siRNA-PABPC1) and siRNA-NC were synthesized by GenePharma. All transfections were performed using Lipofectamine 2000 (Invitrogen).

### Reverse transcription quantitative polymerase chain reaction (RT-qPCR)

Total RNA from cells was extracted using TRIzol Reagent (Invitrogen). Then, the extracted RNA was reverse-transcribed into cDNA using the SuperScript^TM^III First-Strand kit (TOYOBO Co., Ltd., Japan). Subsequently, real-time qPCR was conducted using the SYBR Green PCR Master Mix (Life Technologies, USA) and Stratagene Mx3005P PCR System (Agilent Technologies, USA). The sequences of the primers used are shown in Table 1. U6 was used as the reference for miRNA and glyceraldehyde-3-phosphate dehydrogenase (GAPDH) as that for mRNA. Relative RNA expression was determined using the 2^−ΔΔCt^ method (11).

**Table 1:** Primer sequences used in RT-qPCR.

Gene	Primer sequence (5′-3′)
miR-129-5p	F: GATCCGCAAGCCCAGACCGCAAAAAGTTTTTA
	R: AGCTTAAAAACTTTTTGCGGTCTGGGCTTGCG
PABPC1	F: CACCGGTGTTCCAACTGTTT
	R: TGCTAGACCTGGCATTTGCT
U6	F: AAAGCAAATCATCGGACGACC
	R: GTACAACACATTGTTTCCTCGGA
GAPDH	F: CCCATCACCATCTTCCAGGAG
	R: GTTGTCATGGATGTCCTTGGC

RT-qPCR: reverse transcription quantitative polymerase chain reaction; PABPC1: Poly (A) binding protein cytoplasmic 1; GAPDH: glyceraldehyde-3-phosphate dehydrogenase; F: forward; R: reverse.

### Cell proliferation assay

3-(4,5-dimethylthiazol-2-yl)-2,5-diphenyltetrazolium bromide (MTT), colony formation, and 5-ethynyl-2′-deoxyuridine (EdU) labeling assays were performed to assess cell viability and growth. In the MTT assay, cells were seeded into 96-well plates at 6000 cells/well for 24 h. Then, the cells were treated with PD at different concentrations (0, 5, 10, 20, and 40 µM, diluted in 0.5% FBS-medium) for 72 h. The supernatant was then discarded, and 100 μL MTT solution (1 mg/mL, Sigma-Aldrich Chemical Company) was pipetted into each well. The absorbance at 570 nm was measured using a Spectra Max M5 microplate reader (Molecular Devices, USA). Percent cell viability was determined according to the ratio of the average absorbance of wells treated with PD to that of the treated with DMSO.

In the EdU assay, all experimental procedures were performed using a Cell-Light EdU DNA-replication Assay Kit (RiboBio, China), in strict accordance with the manufacturer's protocols. After the co-incubation of cells with 50 mM EdU for 2 h, the cells were fixed using 4% paraformaldehyde and then stained with Apollo solution and then with Hoechst 33342. The number of EdU-positive cells was counted under a microscope (DMI3000B, Leica, Germany) in five random fields.

In the colony formation assay, cells were seeded on 6-well plates and incubated for 2 weeks. Thereafter, the cells were stained with crystal violet (Solarbio Science & Technology Co., Ltd., China) and observed under an inverted phase-contrast microscope (Axiovert 200, Zeiss, Germany).

### Western blot analysis

Cells were lysed in cold radioimmunoprecipitation assay buffer to collect cell lysates. Then, the total protein and target protein concentrations were determined using the bicinchoninic acid (BCA) method. Protein samples were loaded at equal volumes and electrophoresed in 10% SDS-PAGE and were then transferred onto polyvinylidene fluoride (PVDF) membranes (EMD, Millipore Corp., USA). Thereafter, the membranes were incubated with primary antibodies at 4°C overnight, washed with tris-buffered saline with Tween^®^ 20, and incubated with secondary antibodies for 2 h at room temperature. Subsequently, enhanced chemiluminescence (ECL) reagent was added to the membrane. Protein bands and band intensities were imaged and analyzed using GelPro ANALYZER (Media Cybernetics, USA ), with GAPDH as the internal reference. The antibodies used were as follows: primary antibodies against cleaved caspase-3 (1:1000, #9661, Cell Signaling Technology, USA), B-cell lymphoma-2 (Bcl-2, 1:2000, ab182858, Abcam, Inc., UK), Bcl-2-associated X (Bax, 1:5000, ab32503, Abcam), GAPDH (1:10,000, ab181602, Abcam), PABPC1 (1:1000, ab6125, Abcam), phosphatidylinositol-3 kinase (PI3K, p85 beta, 1:2000, ab180967, Abcam), p-PI3K (p85 beta, Y464, 1:750, ab138364, Abcam), protein kinase B 1 (AKT 1, 1:1000, ab126811, Abcam), and p-AKT1 (s473, 1:7500, ab81283, Abcam). The secondary antibodies were goat anti-rabbit IgG H&L (HRP) (1:20,000, ab6721, Abcam) and goat anti-mouse IgG H&L (HRP) (1:10,000, ab205719, Abcam).

### Cell apoptosis assay

To measure cell apoptosis, we performed Hoechst 33342 (MedChemExpress Co., Ltd., USA) staining and flow cytometry. Cell suspensions were mixed into a single suspension, placed on sterile slides, and observed under a microscope. After the adherence of cells, the cells were treated with different concentrations of PD and incubated for 48 h. Then, the cell slides were fixed in paraformaldehyde, washed, and stained with Hoechst 33342 in the absence of light and at room temperature. The slides were imaged using a fluorescence microscope (Nikon Instruments Co., Ltd., China), and cells were counted in five randomly selected fields. Apoptosis was evaluated using the following formula: apoptosis rate (%) = apoptotic cells/total cells ×100%.

For flow cytometry, the Annexin V-fluorescein isothiocyanate (FITC) cell apoptosis kit (Bestbio Biotechnology Co., Ltd., China) was used. Forty-eight hours after transfection, cells were detached using trypsin and washed with phosphate buffered saline. Thereafter, the cells were resuspended in 1X binding buffer at 1×10^5^ cells/mL. Subsequently, 5 μL Annexin V-FITC and 5 μL propidium iodide were added to the 100 μL cell suspension, and the suspension was incubated for 15 min in the absence of light. Finally, the samples were treated with 400 μL 1X binding buffer, and the apoptosis of cells was determined using the Cell-Quest software (Becton Dickinson, USA) and a flow cytometer (FACSCalibur, Becton Dickinson).

### miRNA microarray analysis

Total RNA was collected using TRIzol Reagent and was purified using the RNeasy Mini Kit (Qiagen, USA). Then, the synthesized cDNA was hybridized using miRNA Expression Microarray (Arraystar, USA). miRNAs with differential expression were screened using the GeneSpring GX v12.1 software package (Agilent Technologies, USA), with P<0.05 and |Log FC| ≥2 set as the screening parameters.

### Luciferase assay

The sites for binding between miR-129-5p and PABPC1 were predicted using StarBase (http://starbase.sysu.edu.cn/) (12). The wild type (WT) PABPC1 fragment containing the putative binding sites of miR-129-5p was subcloned into the pmirGLO vectors (Promega Corp., USA) that was named PABPC1-WT; a mutant type (MT) PABPC1 fragment containing a mutant binding site for miR-129-5p was subcloned into the pmirGLO vector that was named PABPC1-MT. The constructed vectors were co-transfected with miR-129-5p mimic or mimic control into cancer cells. After 48 h, luciferase activity was assessed using a Dual Luciferase Reporter system (Promega).

### Statistical analysis

Data are reported as means±SD. Statistical differences were compared using one-way or two-way analysis of variance followed by Tukey's multiple comparisons test. All data were analyzed using SPSS 22.0 (IBM, USA). P<0.05 was considered statistically significant.

## Results

### PD treatment effectively inhibited bladder cancer cell development

The chemical structure of PD is shown in Figure 1A. The MTT assay results indicated that the viability of cancer cell lines, especially T24, was significantly decreased by PD treatment in a concentration-dependent manner (Figure 1B). On the contrary, PD did not significantly affect the viability of SV-HUC-1 cells, indicating that PD had a selective toxicity towards different bladder cancer cells.

**Figure 1:** Platycodin D (PD) treatment effectively inhibits bladder cancer cell development. **A**, Chemical structure of PD (C_57_H_92_O_28_, M.W. 1225). **B**, Bladder cancer cell lines (T24 and 5637) and human uroepithelial cell line (SV-HUC-1) were treated with different doses of PD (0, 5, 10, 20, and 40 µM, respectively), and the cell viability was determined using the MTT assay 48 h later (*P<0.05 compared to SV-HUC-1 cells, two-way ANOVA). **C**, Protein levels of cleaved caspase-3, Bax, and Bcl-2 in cells were determined by western blot analysis (*P<0.05 compared to 0 µM PD treatment, one-way ANOVA). **D**, Apoptosis rate of cells was determined by Hoechst 33342 staining (scale bar: 200 μm). *P<0.05, **P<0.01 compared to 0 µM PD treatment (one-way ANOVA). Data are reported as means±SD. Three independent experiments were performed.

Furthermore, we explored the role of PD in bladder cancer cell apoptosis. Western blot analysis indicated that, compared to the 0 μM PD treatment, high concentrations of PD resulted in a significant increase in cleaved caspase-3 and Bax levels and a decline in the Bcl-2 level (Figure 1C). Likewise, Hoechst staining indicated that treatment with high concentrations of PD increased the cell apoptosis rate (Figure 1D); the cell apoptosis rate was higher in T24 cells than in 5637 cells. These results indicated that PD can suppress the development and growth of bladder cancer cells, with the T24 cell line having a relatively higher sensitivity to PD.

### miR-129-5p was partially responsible for PD-mediated cancer inhibition

Recently, the dysfunction of miRNAs has been demonstrated to regulate multiple cellular signaling pathways, thereby involving a variety of biological processes (13 [Bibr B14] [Bibr B15]–16). Moreover, miRNA-associated regulatory mechanisms play important roles in various health problems, including bladder cancer (17,18). Thus, to explore the molecular mechanisms involved in miRNA profiles, the T24 cell line, with a strong sensitivity to PD treatment, was used for miRNA microarray analysis. Seventy-two hours after treatment of cells with 40 µM PD, the miRNAs showing differential expression in cells before and after PD treatment were screened (Figure 2A). miR-129-5p, which was found to have the highest expression, was selected for further research.

**Figure 2:** miR-129-5p is partially responsible for platycodin D (PD)-mediated cancer inhibiting events. **A**, Top 10 differentially expressed miRNAs before and after 40 µM PD treatment were analyzed by miRNA microarrays. **B**, miR-129-5p expression in bladder cell lines (T24 and 5637) and human uroepithelial cell line (SV-HUC-1) was determined by RT-qPCR (**P<0.01 compared to SV-HUC-1 cells, one-way ANOVA). **C**, miR-129-5p expression in bladder cancer cells after miR-129-5p inhibitor or inhibitor control transfection was determined by RT-qPCR. **D**, Proliferation of cells was determined by EdU labeling assay (scale bar: 200 μm). **E**, Apoptosis rate of bladder cancer cells was determined by flow cytometry. *P<0.05 (one-way ANOVA). Data are reported as means±SD. Three independent experiments were performed.

We explored the expression of miR-129-5p in T24, 5637, and SV-HUC-1 cells using RT-qPCR. The results indicated that miR-129-5p expression was decreased in cancer cell lines (Figure 2B). To validate the involvement of miR-129-5p upregulation in PD treatment, we further transfected a miR-129-5p inhibitor and an inhibitor control into the cancer cell lines. Twenty-four hours later, the cells were further treated with 40 µM PD and incubated for another 24 h. The cells that were neither transfected nor treated were defined as the blank group, whereas the cells treated with PD were defined as the control group. We found that miR-129-5p expression was successfully downregulated by the miRNA inhibitor (Figure 2C). The EdU labeling assay indicated that the inhibitory effect of PD on bladder cancer cell proliferation was partially blocked by the miR-129-5p inhibitor (Figure 2D). In addition, flow cytometry indicated that the promotion of bladder cancer cell apoptosis by PD was partially inhibited by the miR-129-5p inhibitor (Figure 2E). These findings indicated that miR-129-5p was involved in the inhibition of PD-mediated cancer.

### miR-129-5p directly targeted PABPC1

The binding between miR-129-5p and PABPC1 is shown in Figure 3A. PABPC1 has previously been reported as an oncogene (19). The RT-qPCR and western blot assay indicated that the mRNA and protein expression of PABPC1 was increased in cancer cell lines (Figure 3B). The transfection efficacy of pcDNA-PABPC1 into bladder cancer cells was validated using RT-qPCR (Figure 3C). The colony formation assay (Figure 3D) revealed that cell proliferation was promoted, whereas flow cytometry (Figure 3E) revealed that cell apoptosis was decreased with pcDNA-PABPC1 administration.

**Figure 3:** miR-129-5p directly targets PABPC1. **A**, Targeting between miR-129-5p and PABPC1 predicted using StarBase (http://starbase.sysu.edu.cn/). **B**, mRNA and protein expression of PABPC1 in bladder cell lines (T24 and 5637) and a human uroepithelial cell line (SV-HUC-1) were determined by RT-qPCR and western blot analysis, respectively (*P<0.05 compared to SV-HUC-1 cells, one-way ANOVA). **C**, PABPC1 expression in bladder cancer cells after pcDNA-PABPC1 transfection was determined by RT-qPCR. **D**, Colony formation ability of cells was determined by colony formation assay. **E**, Apoptosis rate of bladder cancer cells was determined by flow cytometry. **F**, miR-129-5p expression after miR-129-5p mimic transfection was determined by RT-qPCR. **G**, mRNA and protein expressions of PABPC1 in cancer cells after miR-129-5p mimic transfection were determined by RT-qPCR and western blot analysis, respectively. **H**, Relative luciferase activity in cells after co-transfection of PABPC1-WT/MT vector and miR-129-5p mimic/mimic control. Data are reported as means±SD. *P<0.05 (one-way ANOVA). Three independent experiments were performed.

To confirm the binding between miR-129-5p and PABPC1, miR-129-5p mimic and the corresponding control were transfected into bladder cancer cells (Figure 3F). RT-qPCR and western blot assay revealed that miR-129-5p mimic significantly inhibited PABPC1 expression (Figure 3G). The direct binding between miR-129-5p and PABPC1 was validated using a dual luciferase reporter gene assay. The PABPC1-WT vector containing the binding site for miR-129-5p and the PABPC1-WT vector containing a mutant binding site for miR-129-5p were co-transfected with miR-129-5p mimic or mimic control into cancer cells. After the co-transfection, decreased luciferase activity was observed in the cells co-transfected with PABPC1-WT and miR-129-5p mimic, whereas no significant changes in luciferase activity were observed in the other co-transfected cells (Figure 3H). These findings validated that miR-129-5p can directly bind to PABPC1.

### PABPC1 activated the PI3K/AKT pathway

A paralogue of PABPC1 and PABPC1L was found to activate the PI3K/AKT signaling pathway and promote the malignant behaviors of colorectal cancer cells (20), as the PI3K/AKT signaling pathway is well-known to play important roles in cancer progression. Hence, we speculated that PABPC1 possibly promotes bladder cancer cell growth through the PI3K/AKT pathway. We transfected pcDNA-PABPC1 or siRNA-PABPC1 or the corresponding NC into cancer cell lines and western blot analysis indicated that PI3K and AKT phosphorylation was significantly increased by pcDNA-PABPC1 but suppressed by siRNA-PABPC1. The total levels of PI3K and AKT exhibited little change (Figure 4).

**Figure 4:** PABPC1 increased phosphorylation of PI3K/AKT. Total PI3K/AKT and phosphorylation of PI3K/AKT determined by western blot analysis. The quantification of PABPC1 expression, PI3K phosphorylation, PI3K expression, AKP phosphorylation, and AKT expression are presented in the graphs. Data are reported as means±SD. Three independent experiments were performed. *P<0.05 (one-way ANOVA).

### PD inhibited bladder cancer progression through the miR-129-5p/PABPC1/PI3K/AKT axis

Twelve hours after the treatment of bladder cancer cells with miR-129-5p inhibitor, the cells were further treated with 40 µM PD for another 24 h. The cells that were neither transfected nor treated were defined as the blank group, whereas the cells treated with PD were defined as the control group. RT-qPCR results indicated that treatment with PD led to a notable decline in the expression of PABPC1 in cells and then the miR-129-5p inhibitor partially blocked this decline (Figure 5A). Western blot analysis showed that the protein levels of PABPC1 and the phosphorylation of PI3K and AKT in cells were inhibited by PD but returned to normal levels after the administration of miR-129-5p inhibitor (Figure 5B). These findings revealed that PD inhibited the PABPC1/PI3K/AKT axis through miR-129-5p.

**Figure 5:** Platycodin D (PD) inhibited bladder cancer progression through the miR-129-5p/PABPC1/PI3K/AKT axis. **A**, PABPC1 expression in cells after PD treatment and miR-129-5p inhibitor pre-transfection was determined by RT-qPCR. **B**, Protein level of PABPC1 and the phosphorylation of PI3K and AKT after PD treatment and miR-129-5p inhibitor pre-transfection were determined by western blot analysis. Data are reported as means±SD. Three independent experiments were performed. *P<0.05 (one-way ANOVA).

## Discussion

Bladder cancer is the most prevalent cancer of the urinary system and a great health concern, with unfavorable treatment outcomes owing to the limited efficacy of current approaches and the complexity of the disease (21). Thus, a greater understanding of the mechanisms underlying bladder cancer and the development of novel therapeutic modalities are required. The present study revealed that PD had a suppressive role in bladder cancer proliferation and that PD was potentially involved in the upregulation of miR-129-5p, the subsequent downregulation of PABPC1, and thereby the inactivation of the PI3K/AKT signaling.

In addition to cough and phlegm reduction, traditional Chinese herbal medicines with phlegm-eliminating properties have been shown to play anti-cancer roles that are primarily attributed to their apoptosis-inducing and proliferation-, invasion-, and migration-inhibiting functions (22). Here, we initially found that PD treatment led to a significant decline in the proliferation of the T24 and 5637 bladder cell lines relative to that of the SV-HUC-1 cell line in a dose-dependent manner and that PD promoted the apoptosis of T24 and 5637 cells. Specifically, PD was shown to trigger the apoptosis of cancer cells via multiple mechanisms, such as Fas/FasL upregulation, mitochondrial impairment, ROS regeneration, Bcl-2 family modulation, apoptosis-inhibitor suppression, and activation of apoptosis-related pathways, such as mitogen-activated protein kinase and the inhibition of pro-survival pathways, including PI3K signaling (5). Experimentally, PD has been demonstrated to induce apoptosis and autophagy in hepatocellular carcinoma cells (23). Likewise, the inhibitory and inductive functions of PD towards the proliferation and apoptosis, respectively, of non-small lung cancer cells have been reported (24). Similarly, the induction of cancer cell death by PD has also been reported to occur through cytoplasmic pinocytic and autophagic vacuolation (25). Collectively, these results revealed the inhibitory role of PD in bladder cancer cell growth.

Based on the findings mentioned above, we further investigated the molecules possibly involved in the anti-cancer effects of PD. Recent research has revealed the important involvement of miRNAs in the therapeutic effects of traditional Chinese medicine on human diseases, including cancer (26,27); the aberrant expression of miRNA during cancer development has also been frequently reported (28,29). A miRNA (miR-34a) has recently been reported to improve the susceptibility of gastric cancer to PD (30), but there is limited information on whether PD alters miRNA expression. Therefore, a miRNA microarray analysis was performed, which identified miR-129-5p as the most upregulated mRNA in cancer cells after high-dose PD treatment. Next, miR-129-5p was found to be poorly expressed in cancer cells relative to the non-PD treated cancer cells; this finding was partly in line with that of a previous report stating that miR-129-5p is poorly expressed in bladder cancer tissues (31). Further experiments suggested that the tumor-suppressing roles of PD were blocked by miR-129-5p inhibitor, indicating that miR-129-5p was at least partially responsible for the anti-cancer function of PD. The tumor-suppressing role of miR-129-5p has been confirmed in gastric cancer (32) and shown to be mediated by the induction of cell apoptosis and repression of cell proliferation and migration. Additionally, miR-129-5p was found to promote sensitivity of bladder cells to gemcitabine therapy, thus promoting cell apoptosis (33).

Next, the online prediction and dual luciferase reporter assay suggested that PABPC1 was a target mRNA of miR-129-5p. PABPC1 was noted as one of the HUB nodes linked to the molecular networks specific for kidney, bladder, and prostate cancers (10). PABPC1 has also been found to be upregulated in superficial bladder cancer tissues (34). Here, we validated the increase in PABPC1 levels in bladder cancer cell lines and found that PABPC1 expression was suppressed after PD but recovered after treatment with miR-129-5p inhibitor. Upregulation of PABPC1 promoted cancer cell growth. These results collectively suggested that PD inhibited bladder cancer growth through the miR-129-5p/PABPC1 axis. In addition, PABPC1L, a paralogue of PABPC1, was found to activate the PI3K/AKT signaling pathway and promote the malignant behaviors of colorectal cancer cells (20). This pathway is well-known to play important roles in cancer progression, including tumor development, growth, proliferation, metastasis, and cytoskeletal reorganization (35). The same therapeutic potential of PI3K/AKT also applies to bladder cancer (36). Here, we identified that pcDNA-PABPC1 significantly increased PI3K/AKT phosphorylation, i.e., PI3K/AKT signaling activation, which suggested that PABPC1 promotes bladder cancer development possibly through the involvement of the PI3K/AKT pathway. As mentioned above, inhibition of the pro-survival pathways, including the PI3K pathway, is potentially responsible for the PD-mediated events (5). Collectively, these findings suggested that PD may suppress bladder cancer development by blocking the PABPC1/PI3K/AKT axis through miR-129-5p.

In conclusion, the present study demonstrated that PD could inhibit bladder cancer growth and development through miR-129-5p and the subsequent PABPC1 downregulation and PI3K/AKT signaling deficit (Figure 6). However, there are still limitations in the present research. Whether PD has a similar cancer-inhibiting role *in vivo* was not studied. In addition, the cancer cell lines used in the current study, T24 and 5637, are p53 mutants. P53 is a tumor inhibitor, and its activation by reactive oxygen species leads to the autophagy and apoptosis of cancer cells (37); however, p53 is always inactivated in tumor cells due to the mutation or deletion of the TP53 gene or inhibited by overexpression of MDM2, leading to metastatic potential (38,39), while PD has been reported to target mutant p53 to suppress the progression of breast cancer (40). Whether PD affects p53 activation and influences reactive oxygen species and autophagy in cancer cells requires further investigation. We plan explore these points as well as the potential functions of PD *in vivo* in future experiments.

**Figure 6:** Molecular mechanism of action. Platycodin D (PD) upregulated miR-129-5p cells to inhibit PABPC1 and reduce the phosphorylation of PI3K and AKT, thus suppressing proliferation while promoting apoptosis of bladder cancer cells.
